# Research on Neck Response of Elderly Drivers in Rear Collision

**DOI:** 10.1155/2022/5239515

**Published:** 2022-06-07

**Authors:** Hequan Wu, Xiaoshun Deng, Lin Hu, Jin Liu, Xiaohao Liu

**Affiliations:** ^1^Key Laboratory and Lightweight and Reliability Technology for Engineering Vehicle, Education Department of Hunan Province, Changsha University of Science and Technology, Changsha 410004, China; ^2^Bioengineering Center, Wayne State University, Detroit 48201, USA

## Abstract

In order to study the neck response of elderly drivers in rear collision, a finite element model for elderly neck was built. By comparing the cadaver experiment data in the literature, the simulation reliability of the head and neck model of the elderly under dynamic load was verified. Through the C-NCAP rear-end collision test on the elderly model, the study showed that the neck of the elderly driver had good dynamic response characteristics. The verified finite element model was used to analyze the head and neck collision response and injury risk of the elderly under different distances between the head and the headrest (vertical distance and horizontal distance). By analyzing the head and neck injuries of occupants at different distances, it was found that when the horizontal distance was 50 mm, and the vertical distance was between +10 and ~+20 mm, the headrest could play the best role in protecting the neck of the elderly driver and could reduce the degree of injury of the elderly driver in the process of rear collision.

## 1. Introduction

With the acceleration of the global aging process, the proportion of elderly drivers has gradually increased in recent years [1]. The most common disabling injuries in accidents included occupant neck injuries [2, 3], which were more likely to occur in the elderly due to intervertebral disc degeneration and osteophytes that compress the cervical spine. Studies had shown that for every year the occupant's age increases, and the probability of life-threatening injuries during a collision increases by 3% [4].

Neck injuries are one of the most common forms of injury in rear-end collisions, and these injuries are usually caused in low-speed collisions. There are various forms of neck injuries, mainly disc injuries, small joint injuries, spinal nerve root injuries, muscle ligament injuries, etc. Injuries to neck ligaments and muscles are mainly caused by overextension of the neck in a rear-end collision [5, 6]. In a rear-end collision, the cervical spine is subjected to shear and axial force from the lateral direction, and adjacent vertebral joints squeeze each other, causing cartilage damage [7, 8]. When the neck is stretched back, the whole body is in an “S” shape, and the instantaneous change in the volume of the spinal cord causes an instantaneous change in pressure, which leads to nerve damage [9].

Head restraints were proposed as a restraint in the 1960s [10] and were shown to be used to reduce head and neck injuries. Since the introduction of head restraints, passenger car occupants had experienced a 9–18% reduction in neck injuries [11]. However, even with headrests in cars, occupant neck injury rates are still high [12]. It may be that the head and headrest position is not adjusted to the correct position resulting in the inability to play a restraining effect on the human head and neck. There had been some studies on the distance between the head and the headrest, and the National Highway Traffic Safety Administration proposed new standards for passenger car seat headrest positions in 2001 [13]. The proposed standard would require all new passenger cars to have headrests that reach a minimum height of 750 mm above the hips when adjusted to the lowest position and 800 mm when adjusted to the highest position. In addition, the horizontal distance from the restraint to the typical seated occupant's head must not exceed 50 mm. The improvement in IIHS ratings proves that manufacturers pay much attention to the distance between the head and the headrest [14]. On the other hand, if the seatback collapses or plastic yields during a rear-end collision, the elastic seatback rebound will be lost or reduced. Several studies had linked seatback collapse to a reduction in the incidence of neck injuries in rear-end collision [15]. Seatbacks showed that some permanent deformation after a crash were less likely to be injured than seats that collapse or did not yield at all. Saab Active Head Restraint (SAHR) was the first application of a series of seatback design measures designed to reduce the risk of injury in rear-end crashes [16]. Active head restraints were designed to move the headrest up and forward, thereby supporting the head before the relative motion between the head and torso became significant. When the load from the occupant was reduced, it returned to its original position. Active headrests further reduced the gap between the head and headrest during a collision, and this reduced force also reduces the risk of thoracic spine injury during a collision, which may be important for reducing S-shaped neck flexion. However, active headrests are still only present in a limited number of cars, and the actual position of the headrests may be somewhat different from the ideal position, which can only reduce the injury of most people. It protects the elderly occupants from neck injuries in rear-end collisions which is limited.

These studies consistently demonstrate the effect of headrest position on occupant head motion response and injury. In volunteer experiments, headrest position significantly affected the size and timing of peak head and chest movements [17]. Changing the headrest backrest can significantly affect the forces and moments at the top and bottom of the neck, as well as the head acceleration and angle. Kitagawa et al. [18] reported that for backrests smaller than 50 mm, no S-shaped bending occurs in the neck region. A human finite element (FE) model was conducted to evaluate the effectiveness of a fixed headrest system with respect to neck injury criteria (NIC) and joint capsule strain. The results of Svensson et al. [19] confirmed that forward positioning of the headrest to reduce the headrest contact time and thus the relative motion between the head and torso contributed to the reduction of neck injury values and joint capsule strain. There had been a lot of studies on the position of car headrest, but the research on elderly occupants was not enough, and there were still many areas to explore. The difference between this study and other studies was that the elderly human model is used to analyze the headrest distance.

A finite element (FE) model of human body and dummy are usually used to study the biomechanical response of the neck under a car collision [20]. In recent years, many representative FE models of human body biomechanics have been developed [21, 22], which excludes elderly body models. Kleinberger [23] used the MADYMO whole-body model to study the effect of changing the headrest backrest from 0 to 152 mm on the human body. And they analyzed the relative motion between the head and upper thorax (T1), the forces and moments at the level of the atlanto-occipital joint, and the injury criteria. There were some studies that analyzed the behavior of different drivers [24–27] but less analysis of older drivers. The establishment of the FE model of the elderly body was very complicated. Due to the increase of age, the water and bone minerals in the nucleus pulposus of the elderly will be partially reduced, and the elasticity will be significantly reduced. In the elderly, the intervertebral space will become narrower, resulting in lower injury tolerance during collisions. Therefore, it is necessary to consider establishing a FE model that can represent the elderly body for research on occupant protection.

In this study, we analyzed the damage response of the FE model of the neck of the elderly and compared it with related cadaver experiments. This study investigated the biomechanical response to neck injuries of elderly drivers at different distances (horizontal distance and vertical distance) between the head and the headrest during a rear-end collision.

## 2. Materials and Methods

### 2.1. Establishment of Neck Geometry Model and Material Parameters

This article used an FE model of the neck and head of the elderly which was established at the Wayne State University (WSU) and Toyota Safety Research Center. The specific modeling process is shown in Figure 1. In the development of the finite element model of the elderly body, the material parameters of the components in the model were determined by the relevant researchers at the Wayne State University Bioengineering Center using the following methods: for the hard skeletal tissues of the human body, the vast majority have elastic-plastic properties, and for the soft tissues of the human body, they are usually defined as nonlinear materials or viscoelastic materials. Using the study of relevant literature, tissue materials related to the elderly body at home and abroad are discovered and directly applied to this model; while for material parameters that are difficult to obtain or specific to human body characteristics, they can be calculated by scaling according to the functional relationship between the human body and the corresponding tissue material parameter models established in the literature. The final elderly body needs to be reevaluated and determined based on the data from each validation experiment. The skeletal structure in the model used in this study was mainly meshed with hexahedral elements (cancellous bone) and shell elements (cortical bone). For the ligaments between the cervical vertebrae, 1D linear elements that only bear tension were used to model the ligaments as shown in Figure 2. The bone model used elastic-plastic materials, and muscles were defined as viscoelastic materials; ligaments and cartilage were defined as elastic materials, and the FE model materials of the neck [28] were shown in Table 1. The threshold of neck injury adopts the threshold obtained from the cadaver test in the literatures [29–31], as shown in Table 2.

Based on the statistical model in the literature, we adjusted the skeletal angle of the neck and head, and the chord angle of the neck is 78.9 degrees, as shown in Figure 3(a). The FE model of the neck had a complete anatomical structure. It is usually divided into three parts: the upper cervical spine (C1 and C2), the middle cervical spine (C3-C5), and the lower cervical spine (C6-C7), as shown in Figure 3(b) .

### 2.2. Verification of the Finite Element Model

In order to obtain the biomechanical response of the neck of the elderly under dynamic load, we referred to the axial impact experiment of Nightingale et al. [33] to apply a load to the head and neck of the cadaver, as shown in Figure 4(a) .  Table 3 listed the collision boundary conditions and damage of these corpse samples.

According to the cadaver test data, the elderly head and neck model was verified. The simulation setup is shown in Figures 4(b) and 4(c). Loaded mass point 16 kg at T1 of the head and neck model to simulate effective torso mass. The initial collision velocity was set to 3.14 m/s in order to be consistent with the cadaveric experiment. The foam plane was simulated by a plastic sheet at the bottom of a cylindrical foam liner. The rigid plane was simulated by a plastic sheet attached to the rigid plate. Six groups of experimental data were selected from 22 experimental samples as the comparative data for model validation, as shown in Table 3. The distance between the head and the pad was set at 1 mm; the contact friction coefficient was 0.2, and the degree of freedom of thoracic T1 was constrained. The sensor position was also the same as in the test. The damping is 0.04, and the energy profile of the head impacting the object is shown in Figure 5. The energy of the rigid impact in Figure 5(a) is mainly concentrated in the first 10 ms, and the energy is much larger than that of the foam impact. The energy of foam impact in Figure 5(b) was mainly concentrated in the first 20 ms, and the energy curve decreased gradually at the moment of head rebound.

The common injury evaluation standard is NIC (neck injury criterion), proposed by Boström et al. [34], and the formula is as follows:

(1) $$\begin{array}{c} \text{NIC}={\upsilon_{rel}}^{2}+0.2\times a_{rel},\\ a_{rel}={a_{x}}^{T1}-{a_{x}}^{Head},\\ v_{rel}=\int_{0}^{t}a_{rel}dt. \end{array}$$

*a*_*x*_^*T*1^is the acceleration in the*x*direction of T1,*a*_*x*_^*Head*^is the acceleration in the*x*direction of the head's center of gravity,*a*_*rel*_is the relative acceleration, and*v*_*rel*_is the relative horizontal velocity of the upper and lower ends of the neck, assuming that the maximum value of the NIC from the start of the rear collision to the time when the head and the headrest are in contact is NIC_max_ and the threshold of NIC_max_ is 15 m^2^/s^2^.

The angle of the impact surface was varied between -15° (posterior head impact) and +15°(anterior head impact). The response of the elderly human head and neck model was carried out in the plane ±15° as shown in Figure 6, and the kinematic response is shown in Figure 7.

In the 0° rigid impact simulation experiment, the overall motion response of the head and neck is shown in Figure 7(a). The head and neck began to contact the pad at 0 ms. At 15 ms, when the head compressed downwards of the rigid plate, the neck deformed and the stress concentrations at the junction of C7 and T1. The pad compressed to the minimum at 21 ms. At this point, the upper cervical spine was in the flexion stage, while the lower cervical spine is in the extension stage, and the neck as a whole was S-shaped spinal curvature. Between 21 ms and 33 ms, the head rebounded and rose, and between 33 ms and 60 ms, the head left the rigid pad. In the 0° foam impact simulation test, the head touched the pad at 0 ms, the head and neck compressed the pad to the lowest at 21 ms, and the neck stress reached the maximum at 31 ms. At 60 ms, the head rebounded and rose as shown in Figure 7(b). Compared with the rigid impact, the flexion deformation of the cervical spine was smaller with the foam impact. In the +15° foam impact test, after 26 ms, the upper cervical spine showed a smaller flexion mode, while the lower cervical vertebra presented an extension pattern, and the whole cervical vertebra presented an S-shaped deformation. Compared with the 0° foam impact, the forward movement of the head in the +15° foam impact test was relatively large. And the overall stress distribution of the head and neck is shown in Figure 7(c).

In the -15° foam impact test, the head was subjected to backward force and moved backward, resulting in the overall buckling deformation of the cervical spine. The mechanical response of head and neck motion is shown in Figure 7(d). Compared with rigid impact, the neck deformation and neck stress of foam impact are smaller.

Table 4 shows the injury data of the head and neck of the elderly under different impact angles and pads. By analyzing the data in Table 4, the head force of the elderly human model was basically within the range of the cadaver experiment. In the rigid plate, the neck force of the model was similar to that of the corpse experiment. However, in the foam plate, the force on the neck of the model was less than that in the corpse test, which may be caused by the difference in head shape and test errors.

Figure 8(a) shows the comparison between the head contact force and the cadaver test curve in the simulation process of rigid plate impact. It can be seen that the overall variation trend of the simulation test curve and the cadaver test curve was basically the same, within the upper and lower boundary curve. The slight difference was that the peak of the simulated curve appeared earlier than the peak of the cadaver test curve. It was caused by the fact that the start time of simulation test was earlier than that of cadaver test.  Figure 8(b) shows the comparison between the head contact force under foam plate impact and the corpse experiment. The action of the head force with time may be related to the action of the skin of the head and the muscles of the head resulting in two-phase [35]. From the overall force trend, the peak time appeared later than the corpse experiment, which due to the difference between the age samples is used in the simulation and the experiment. The experimental samples of cadaver were older, and the tissue structure changes. The head force of the simulation experiment was basically within the upper and lower boundary curve of the corpse experiment. The elderly human head model is able to simulate the head impact response, and the validation of the model is considered effective under this condition.

### 2.3. Global Model Validation

An overall rear crash study of the neck of an elderly FE model was conducted with reference to the rear crash test of the New Vehicle Evaluation Protocol 2018 edition [36]. The authors conducted a study using a commercial car seat model downloaded from the official website. And the introduction of the seat belt system (pretensioner, winder, and slip ring) is in order for the elderly. The part in contact with the human body consists of 2D elements, which are described using the fabric propriety model and 1D elements (seat belt propriety model). The sliding of the seat belt is defined by setting up a slip ring. The skeleton of the seat and the floor are modeled as rigid bodies. During the analysis, all other elements are considered “deformable.” In the course of the study, the authors tried to investigate the overall motion response of the elderly in postcrash. According to the vehicle acceleration curve obtained from the rear-end collision test, it is loaded on the rigid seat and used to simulate the car rear-end collision experiment; the curve corresponds to a collision speed of 20 km/h. The final system is shown in Figure 9.

Figure 10 showed the movement process of the elderly human model under C-NCAP (rear-end collision test). During the 0-40 ms process, the chest of the elderly driver is pushed forward by the seat backrest, but at this time the occupant's head is not in contact with the seat due to inertia to maintain the original position, the upper cervical spine is flexed forward, and the lower cervical spine is extended backward. Due to the tangential force of the cervical spine on the head, the head turns backward, the whole cervical spine extends backward, and the head contacts the headrest. At 40-55 ms, the backward motion continues due to inertia. In 55-65 ms, the energy stored in the seat is transferred to all parts of the body, so that the head produces forward rebound movement, and 65 ms-145 ms when the occupant in the seat belt under the action of the head and neck forward movement.

From the cervical spine stress distribution in Figure 11, it can be seen that the stress was concentrated at C3, which might be due to the fact that the entire cervical spine stretches backward and the head touches the seat at 40 ms. Local stress was high at the C2 and C3 interconnects.

Table 5 shows the magnitude of injury to the neck of the elderly model under the C-NCAP test. It can be seen that the neck of the elderly was subjected to a relatively large tensile force and was subjected to smaller shear and torque. The neck injury value NIC did not exceed the threshold value of 15 m^2^/s^2^, which indicates that neck injury does not occur in the elderly at this collision speed. The experimental results showed that the elderly driver model could simulate the real human body movement during the whole loading.

### 2.4. Parametric Study

Morris et al. [37] reported the use of head restraints in rear impact to reduce the chance of excessive injury to the cervical spine. The horizontal distance between the head and the headrest was defined as the horizontal distance between the last position of the head and the front plane of the headrest, and the vertical distance between the head and the headrest was defined as the vertical distance between the apex of the head and the upper plane of the headrest, as shown in Figure 12(a). The IIWPG (International Insurance Whiplash Prevention Group) and Euro NCAP measured the head and headrest position [14] and then classified the distance between the head and the headrest into four classes, as shown in Figure 12(b), with the above definitions in side view.

According to the position of the headrest scoring grade, the horizontal position of the head from the headrest is mainly between 0 and 100 mm, and the vertical position of the head from the headrest is mainly between 0 and 120 mm. Stemper et al. [17] showed that the horizontal position of the head from the headrest should preferably be controlled within 60 mm, and if it exceeds 60 mm, overextension of the neck would occur. Garcia and Ravani [38] reported that for an initial horizontal distance of less than 50 mm between the head and the headrest, no S-shaped flexion occurs in the cervical region. In this paper, according to the above study, the vertical distance of the head from the headrest is set to 0 mm, and the horizontal distance of the head from the headrest is set to 0–80 mm. Set the postcrash speed to 20 km/h, set the simulation duration to 150 ms, and import LS-DYNA software for calculation. The headrest model was downloaded from the official website of LS-DYNA.

After finding the optimal horizontal distance between the head and the headrest, the best vertical distance between the head and the headrest was studied under this condition. According to the position scoring grade of the headrest, the vertical distance between the headrest and the head is set to ±10 mm, ±20 mm, ±30 mm, ±40 mm, and ±50 mm between -50 and+50 mm for 10 working conditions in the upward direction as the positive direction, as shown in Figure 13, keeping the horizontal distance between the head and the headrest at 50 mm.

## 3. Results and Discussion

Based on the cadaver experiments, this paper established a biomechanical finite element model of the head and neck of the elderly. The head and neck model of the CHARM-70 was evaluated for damage under three different angles (0°, +15°, and -15°) and two different collision planes (rigid plane and foam plane). Under the same constraints, compared with the experimental data of Nightingale et al. [33], the kinematic response and experimental results of the elderly body model and the cadaver test had appealed a higher degree of matching. The elderly body neck model had good lifelikeness. Finally, under the same rear impact speed, the collision damage study under different distances between the head and the headrest (vertical distance and horizontal distance) was carried out, and the results and response of head and neck tissue damage were analyzed.

Table 6 provides statistics on the magnitude of neck injury for elderly occupants at different horizontal distances for a vertical distance of 0 mm between the head and the headrest. When the horizontal distance was 0 mm, the peak acceleration of the head mass of the elderly driver was the largest. At a horizontal distance of 50 mm, the maximum cortical bone stress and the peak acceleration of the head mass of the elderly were smaller. In summary, the optimal headrest and head horizontal distance was 50 mm.

According to Table 7, when the horizontal distance between the head and the headrest was certain (50 mm), and the vertical distance between the head and the headrest was 0 to +50 mm, the maximum stress value of the cortical bone in the neck of the elderly occupants is between 380 and 400 MPa, and the maximum value of the peak stress of the cortical bone and the intervertebral disc is at the vertical distance of +50 mm, while the maximum value of the peak stress of the cancellous bone is at the vertical distance of 0 mm.

It can be found that the injury when the position of the headrest is lower from the head is greater than the injury when the position of the headrest is higher from the head. When the vertical distance between the head and the headrest was 0 mm to -50 mm, the cortical bone cancellous bone and disc stress in the neck of the elderly basically increased with the increase of the distance in the negative direction. Overall, when the vertical distance between the head and the headrest is +10 to +20 mm, the headrest can provide better protection. This is different from the literature [39] where the optimal vertical distance between the head and the headrest was 0 mm in middle-aged people.

In the simulation test of different distances between the head and the headrest, the maximum stress of the vertebrae of the elderly model is higher than that of the middle-aged model. The main reason is that the bone density of the elderly cadaver gradually decreases, the bone becomes brittle and easy to fracture. Moreover, the organizational structure of the elderly has also changed, and other parameters will be different from those of middle-aged people.

When the vertical distance between the head and the headrest was constant (0 mm), the horizontal distance changed, and the stress on the cervical intervertebral disc was less than the stress at a horizontal distance of 80 mm. There are three reasons of the increase in the neck force and moment. First of all, the horizontal distance between the head and the headrest is large. Second, the impact speed of the head and the headrest increased. Finally, the impact force received by the head increased. When the horizontal distance was 0 mm, the head was in direct contact with the headrest, and the greater head impact results in greater peak acceleration of the head. When the horizontal distance was 50 mm, the rear end of the head contacts the headrest at an early moment in the backward movement stage of the head, which reduced the backward displacement of the head and the deformation of the neck. When the horizontal distance between the head and the headrest is constant (50 mm) and the vertical distance is negative, the stress of the cortical and cancellous bones of the neck basically increases with the increase of the vertical distance of the head and neck. The main reason was that the vertical distance between the head and the headrest was too low. It was equivalent to setting a new fulcrum on the neck of the headrest, which makes the neck injury more serious [40]. When the height of the headrest was adjusted to be higher than the center of mass of the head (+10~+20 mm), the rear displacement of the head relative to the thoracic spine can be effectively restrained, and the damage during the rear collision was reduced.

## 4. Conclusions

Nowadays, the degree of aging is increasing. It is necessary to study the risk of head and neck injury of the elderly group in the case of a rear collision and the impact of different positions of the headrest.

1. This article first validated the elderly body and neck model CHARM-70. The kinematic response and experimental results of the elderly body head and neck model and the cadaver test had a high degree of matching, which proved that the model could reflect the movement of the elderly body head and neck in mechanical response and stress distribution
2. Used simulation software to simulate the C-NCAP whiplash test to further verify the finite element model of the elderly body. The test results showed that the occupant model could simulate the real human body movement when the whole was loaded
3. To reduce and minimize human neck injuries in road traffic accidents, we analyzed the head and neck injuries of the occupants at different distances. It was found that the horizontal distance between the headrest and the head was 50 mm, and the vertical distance between the head and headrest was +10~+20 mm; the headrest could protect the neck of elderly drivers and reduce the risk of injury in rear collision
4. In future studies, the effects of headrest angle and headrest stiffness on the risk of head and neck injury in older adults in rear-end collisions will be investigated

## Figures and Tables

**Figure 1:** Schematic diagram of the development of the FE model of the elderly body.

**Figure 2:** Schematic diagram of the position of C7 ligament.

**Figure 3:** Schematic diagram of the elderly neck model.

**Figure 4:** Experimental device setup.

**Figure 5:** Energy of head impact.

**Figure 6:** Schematic diagram of impact angle.

**Figure 7:** Mechanical response of neck cushion impact motion of elderly human model.

**Figure 8:** Comparison of simulation and experimental results.

**Figure 9:** Test conditions.

**Figure 10:** Impact response of C-NCAP elderly body model.

**Figure 11:** Stress distribution of rear-end impact.

**Figure 12:** Diagram of simulation test and cadaver test.

**Figure 13:** The vertical distance between the head and the headrest.

**Table 1:** Some material properties of CHARM-70 neck model [32].

Part	Material parameters
Cancellous of neck	*ρ* = 1.09*e*^−6^*kg*∙*mm*^−3^, *E* = 0.29*Gpa*, *γ* = 0.3, *k* = 0.007118, *N* = 0.2741
Cortical of neck	*ρ* = 2*e*^−6^*kg*∙*mm*^−3^, *E* = 16.8*Gpa*, *γ* = 0.3
Cervical disc	*ρ* = 1.36*e*^−6^*kg*∙*mm*^−3^, *K*_*m*_ = 1.72
Spinal nucleus	*ρ* = 1.36*e*^−6^*kg*∙*mm*^−3^, *k* = 1, *N* = 2.*MU* = 0.1
Neck muscles	*ρ* = 1.1*e*^−6^*kg*∙*mm*^−3^, *B* = 0.005, *β* = 3.0*e*^−5^
Neck ligament	*ρ* = 1.2*e*^−6^*kg*∙*mm*^−3^, *k* = 1.8, *TDF* = 13.56*mm*
Neck cartilage	*ρ* = 1.36*e*^−6^*kg*∙*mm*^−3^, *B* = 2.0

Note: *ρ*: density; *E*: Young's modulus; *γ*: Poisson's ratio; *k*: strength coefficient; *N*: hardening coefficient; *B*: elastic bulk modulus; Km: linear bulk modulus; MU: damping coefficient; *β*: attenuation coefficient; TDF: tensile displacement at failure.

**Table 2:** Injury prediction threshold.

Injury standard	3-year old	50-year old	95-year old
Tension tolerance (Yoganandan, 1996)	1430 N	4000 N	5350 N
Compression tolerance (Mertz, 1978)	1380 N	4170 N	4830 N

**Table 3:** Experimental data of head impact on cadaver.

Number	Type	Angle (°)	Body number	Age/years	Velocity/(m/s)	Maximum head force (*N*)	Resultant force of the neck injury (*N*)
1	Foam	0	N02-P	75	3.14	3452	2016
			N-03	75	3.08	5664	3701
2		+15	I11-P	63	3.2	3155	2096
			I04-P	63	3.19	3383	2901
3		-15	NA2-P	61	3.16	4749	2091
			I25-P	59	3.07	5963	3448
4	Rigid	0	N22-R	71	3.26	8111	3010
			N24-R	62	3.20	8566	2643
5		+15	I32-R	78	3.18	8234	2921
			D41-R	69	3.11	8604	3885
6		-15	UK3-R	62	3.13	5093	4084
			N11-R	55	3.14	11621	2891

**Table 4:** Damage data statistics.

Type	Angle/°	Neck force of simulation/*N*	Neck force range of cadaver/*N*	Head force of simulation/*N*	Head force range of cadaver/*N*
Rigid plate	0	2652.6	2643~3010	10354	8111~8566
	-15	2648.6	2891~4084	6975.6	5093~11621
	+15	2471.9	2921~3885	6465.5	8324~8604
Foam plate	0	1158.3	2016~3701	3678	3452~5664
	-15	1118.5	4749~5963	3498.3	3115~3383
	+15	1120.9	2096~2901	3441.5	2604~5963

**Table 5:** Neck injury value of elderly occupants.

Index	CHARM-70	Damage threshold
NIC (m^2^/s^2^)	8.7	15
Upper neck Fx (*N*)	45.8	340~730
Upper neck Fz (*N*)	161.5	475~1130
Lower neck Fx (*N*)	58.9	340~730
Lower neck Fz (*N*)	627.8	257~1480

Note: *Fx*: shear force; *Fz*: tensile force.

**Table 6:** Damage analysis of different horizontal distances between head and headrest.

Horizontal distance/mm	Max stress of cortical/MPa	Max stress of cancellous/MPa	Max intervertebral disc stress/MPa	Peak acceleration of head center of mass/g
0	347.28	6.75	43.1	1.05
10	437	7.41	39.7	0.99
20	442	7.6	41.4	0.92
30	460	7.65	39	0.91
40	455.3	7.62	38.7	0.93
50	384.6	7.66	43.3	0.88
60	390.6	7.53	48	0.81
70	387.67	7.94	56.9	0.86
80	412.1	7.75	61.4	0.82

**Table 7:** Damage analysis of different vertical distances between head and headrest.

Vertical distance/mm	Maximum stress of cortical/MPa	Maximum stress of cancellous/MPa	Maximum intervertebral disc stress/MPa	Peak acceleration of head center of mass/g
+10	385	7.49	43.3	0.868
+20	388.4	7.47	43.4	0.869
+30	390.56	7.44	43.5	0.939
+40	392.6	7.45	43.8	0.9
+50	400	7.41	47.5	0.936
0	385	7.66	43.3	0.88
-10	410.8	7.67	43.4	0.847
-20	418.7	7.67	43.4	0.847
-30	452.4	7.93	43.5	0.814
-40	463.1	7.91	44.1	0.764
-50	478.1	7.68	44.5	0.854

## Data Availability

The FE Model data used to support the findings of this study are included within the article.
